The article "circ_AKT3 knockdown suppresses cisplatin resistance in gastric cancer" was published in 2022. Journal: Open Med (Wars).

# circ_AKT3 knockdown suppresses cisplatin resistance in gastric cancer

**DOI:** 10.1515/med-2021-0355

**Published:** 2022-02-14

**Authors:** Wenting Shi, Fang Wang

**Affiliations:** School of Clinical Medicine, Changchun University of Chinese Medicine, Changchun, Jilin 130117, China; School of Clinical Medicine, Changchun University of Chinese Medicine, No. 1035, Boshuo Road, Changchun, Jilin 130117, China

**Keywords:** gastric cancer, cisplatin resistance, circ_AKT3, miR-206, PTPN14

## Abstract

**Background:**

Circular RNAs (circRNAs) are associated with cisplatin resistance in gastric cancer (GC). This study aims to explore the role of circRNA AKT serine/threonine kinase 3 (circ_AKT3) in the resistance of GC to cisplatin.

**Methods:**

42 sensitive and 23 resistant GC patients were recruited for tissue collection. The cisplatin-resistant GC cells MKN-7/DDP and HGC-27/DDP were used for *in vitro* study. circ_AKT3, microRNA-206 (miR-206) and protein tyrosine phosphatase non-receptor type 14 (PTPN14) levels were detected via quantitative reverse transcription real-time PCR (qPCR) and Western blot. Cisplatin resistance was assessed by detecting P-glycoprotein (P-gp) level, half maximal inhibitory concentration (IC_50_) of cisplatin and cell apoptosis. The target relationship between miR-206 and circ_AKT3 or PTPN14 was analyzed via dual-luciferase reporter and RNA pull-down assays. The role of circ_AKT3 *in vivo* was assessed using xenograft model.

**Results:**

circ_AKT3 level was increased, but miR-206 was declined in cisplatin-resistant GC tissues and cells. circ_AKT3 knockdown or miR-206 overexpression decreased the level of P-gp and IC_50_ of cisplatin and increased apoptosis of MKN-7/DDP and HGC-27/DDP cells. Additionally, circ_AKT3 targeted miR-206, and regulated cisplatin resistance by interacting with miR-206. PTPN14 was regulated by circ_AKT3 through miR-206 as a bridge. Also, circ_AKT3 knockdown decreased xenograft tumor growth.

**Conclusion:**

circ_AKT3 knockdown suppressed cisplatin resistance using miR-206/PTPN14 axis in cisplatin-resistant GC cells.

## 1 Introduction

Gastric cancer (GC) is one of the main malignancies with high mortality and incidence [1]. Surgery is the main therapeutic strategy of GC, while the clinical outcomes of advanced GC patients remain poor. The combined treatment of surgery and chemotherapy or radiotherapy has been implemented in GC [2]. Cisplatin (DDP) is a major known chemotherapy drug, whereas development of drug resistance limits its therapeutic efficacy [3]. Hence, it is necessary to urgently explore novel strategies to improve cisplatin sensitivity in GC treatment.

Noncoding RNAs, such as circular RNAs (circRNAs) and microRNAs (miRNAs), are not able to code proteins and play important roles in development and therapeutics of cancers [4]. circRNAs have a covalently closed continuous loop structure and play essential roles in cancers [5]. Moreover, circRNAs are associated with occurrence of chemoresistance in human cancers [6]. circRNA AKT serine/threonine kinase 3 (circ_AKT3) is derived from AKT3, which has been regarded to have a vital role in glioblastoma and clear cell renal cell carcinoma [7,8]. More importantly, circ_AKT3 could increase chemoresistance in GC by suppressing miR-198 [9]. However, the mechanism involving circ_AKT3 is complicated and requires further investigation, particularly with respect to cisplatin resistance.

miRNAs regulate eukaryotic gene expression and exhibit pivotal roles in diagnosis, therapy and prognosis of GC [10]. Former works suggested that miR-206 could inhibit resistance to drugs, such as paclitaxel, euthyrox, gefitinib and cisplatin [11,12,13,14]. Moreover, miR-206 is reported to play an anti-cancer role and could inhibit cisplatin resistance in GC [15]. Nevertheless, whether miR-206 is responsible for circ_AKT3-meidated cisplatin resistance is unknown. Furthermore, previous studies report that protein tyrosine phosphatase non-receptor type 14 (PTPN14) is an oncogene and associated with drug resistance in GC [16,17]. Through bioinformatics analysis, we found the predicted complementary sites of miR-206 with circ_AKT3 and PTPN14. Thus, we hypothesized that miR-206 and PTPN14 might be associated with the mechanism addressed by circ_AKT3. In this study, we investigated the influence of circ_AKT3 on cisplatin resistance in GC and explored whether it was regulated by miR-206/PTPN14 axis.

## 2 Materials and methods

### 2.1 Patients and tissues

42 cisplatin-sensitive and 23 cisplatin-resistant patients with advanced GC were recruited for this study. Patients had undergone two cycles of cisplatin-based chemotherapy and were divided into sensitive or resistant group according to the efficacy of the therapy [18]. The cancer tissues were collected and stored at −80°C for RNA extraction. Written informed consents were obtained. This study was approved by the ethics committee of the Changchun University of Chinese Medicine.

### 2.2 Cell culture and transfection

MKN-7 and HGC-27 cells were purchased from BeNa Culture Collection (Beijing, China). The corresponding cisplatin-resistant variants MKN-7/DDP and HGC-27/DDP were obtained through exposure to increased doses of cisplatin. All cells were grown in RPMI-1640 medium (Gibco, Carlsbad, CA, USA) containing 10% fetal bovine serum (Gibco). To maintain the resistant phenotype, the resistant cells were cultured in a medium containing 1 μg/mL cisplatin (Sigma, St. Louis, MO, USA).

Small interfering RNA (siRNA) for circ_AKT3 (si-circ_AKT3), negative control (si-NC), circ_AKT3 overexpression vector, pcDNA circRNA mini vector (vector), PTPN14 overexpression vector, pcDNA3.1 empty vector (pcDNA), miR-206 mimic, miRNA negative control (miR-NC), miR-206 inhibitor (anti-miR-206) and inhibitor negative control (anti-miR-NC) were synthesized by RiboBio (Guangzhou, China). Upon reaching 60% confluence, MKN-7/DDP and HGC-27/DDP cells were transfected with 40 nM oligonucleotides or 500 ng vectors via LipoFiter^TM^ Liposomal Transfection Reagent (Hanbio, Shanghai, China) and cultured for 24 h.

### 2.3 RNA isolation and quantitative reverse transcription PCR (RT-qPCR)

RNA isolation was performed through Trizol-based methods. The RNA was employed for reverse transcription and RT-qPCR using All-in-One^TM^ First-Strand cDNA Synthesis Kit and RT-qPCR Detection Kit (FulenGen, Guangzhou, China). The specific primers used in this study were shown as follows: circ_AKT3 (Forward, 5′-TTGGTGGAGGACCAGATGAT-3′ and Reverse, 5′-ATAGAAACGTGTGCGGTCCT-3′); PTPN14 (Forward, 5′-TCTAGGATGTGTGCCAGGGA-3′ and Reverse, 5′-TGTGGTGCTTCCGGAAATGT-3′); and GAPDH (Forward, 5′-ACAACTTTGGTATCGTGGAAGG-3′ and Reverse, 5′-GCCATCACGCCACAGTTTC-3′). The primers for miR-206 and U6 were provided by FulenGen with a universal adaptor PCR primer. The relative expression levels of circ_AKT3, PTPN14 and miR-206 were analyzed according to the 2^−ΔΔCt^ method with GAPDH or U6 as a reference [19].

### 2.4 Cisplatin cytotoxicity assay

Cisplatin cytotoxicity was investigated by a MTT Cell Cytotoxicity Assay Kit (Beyotime, Shanghai, China). MKN-7/DDP and HGC-27/DDP cells (10,000 cells per well) were placed into 96-well plates overnight and then incubated with a series of concentrations (0–20 μg/mL) of cisplatin for 48 h. Then, the cells were incubated with MTT reagent for 4 h and then incubated with formazan dissolving solution. Subsequently, the output of the absorbance at OD570 nm was determined with a microplate reader (Bio-Rad, Hercules, CA, USA). The half maximal inhibitory concentration (IC_50_) of cisplatin was estimated according to the survival curve.

### 2.5 Western blot

MKN-7/DDP and HGC-27/DDP cells were lysed for total protein isolation using RIPA buffer with 1% phenylmethylsulfonyl fluoride (Solarbio, Beijing, China). After the high-speed centrifugation (12,000*g*, 5 min) at 4°C, the protein in supernatant was quantified and used for SDS-PAGE. Transmembrane was performed using nitrocellulose membranes (Solarbio) and western blot transfer buffer (10×, Solarbio). QuickBlock^TM^ Blocking Buffer (Beyotime) was used for blocking the nonspecific binding sites. Subsequently, the membranes were incubated with primary antibodies overnight and then interacted with special secondary antibody. The antibodies against p-glycoprotein (P-gp) (ab235954), PTPN14 (ab204321), GAPDH (ab181602) and immunoglobulin G (ab205718) were obtained from Abcam (Cambridge, MA, USA). Protein signals were developed using BeyoECL Plus (Beyotime). The relative protein expression was half-quantified with Quantity One software (Bio-Rad) and normalized to GAPDH level.

### 2.6 Cell apoptosis assay

Cell apoptosis was measured through flow cytometry using an Annexin V-fluorescein isothiocyanate (FITC)/propidium iodide (PI) apoptosis detection kit (Solarbio). MKN-7/DDP and HGC-27/DDP cells (100,000 cells per well) were added into 6-well plates and cultured for 48 h. Subsequently, cells were incubated with 10 μL of Annexin V-FITC and PI. The apoptotic rate was determined using a flow cytometer (Agilent, Hangzhou, China) displaying the percentage of cells labelled by Annexin V-FITC + and PI +/−.

### 2.7 Bioinformatics analysis, luciferase reporter analysis and RNA pull-down

Bioinformatics analysis was used to search potential binding sites of miR-206 and circ_AKT3 or PTPN14 by using starBase. For luciferase reporter assay, firefly luciferase-expressing pmirGLO vectors (Promega, Madison, WI, USA) were exploited for establishment of wild-type (Wt) or mutant (Mut) luciferase reporter vectors targeting circ_AKT3 or PTPN14, named as circ_AKT3-Wt, circ_AKT3-Mut, PTPN14 3′UTR-Wt or PTPN14 3′UTR-Mut, respectively. MKN-7/DDP and HGC-27/DDP cells were co-transfected with miR-206 mimic or miR-NC and these constructs, along with renilla vector. After 24 h post-transfection, luciferase activity was detected through a luciferase reporter assay kit (Promega).

For RNA pull-down, the Wt or Mut sequences of miR-206 and circ_AKT3 were labeled with biotin, and named as bio-miR-206, bio-miR-206-Mut, bio-circ_AKT3 and bio-circ_AKT3-Mut, respectively. The bio-miR-NC and bio-NC were used as the control. MKN-7/DDP and HGC-27/DDP cells were lysed in RIPA buffer with RNase inhibitor (Invitrogen, Carlsbad, CA, USA) and then incubated with biotinylated products for 2 h, followed by incubation with streptavidin beads for 1 h. After extraction of bound RNAs, the expressions of circ_AKT3 and miR-206 enriched in precipitates were detected by RT-qPCR analysis.

### 2.8 Xenograft model

The 5-week-old male BALB/c nude mice were obtained from Beijing Laboratory Animal Center (Beijing, China). The lentiviral vector of short hairpin RNA targeting circ_AKT3 (sh-circ_AKT3) or negative control (sh-NC) was generated by RiboBio. MKN-7/DDP cells (2 × 10^6^ cells per mouse) stably transfected with sh-circ_AKT3 or sh-NC were subcutaneously injected into the flanks of the mice (*n* = 6/group). Tumor volume was examined every 4 days after 7 days and calculated as: 0.5 × length (mm) × width^2^ (mm^2^). After 31 days, the mice were killed by cervical dislocation. Tumor weight was measured and tumor samples were collected for the abundances of circ_AKT3, miR-206, PTPN14 and P-gp. The animal experiments were approved by the Animal Care and Use Committee of the Changchun University of Chinese Medicine.

### 2.9 Statistical analysis

Statistical analysis of every experiment was conducted by GraphPad Prism 6 (GraphPad Inc., La Jolla, CA, USA). The data from three independent experiments were shown as mean value ± standard deviation. Student’s *t* test or Mann-Whitney test was employed for the comparison between the two groups, while ANOVA with Tukey test was employed for the comparison between three or more groups. The potential linear relationship between miR-206 and circ_AKT3 or PTPN14 level was analyzed by spearman’s correlation assay. *P* < 0.05 was considered as significant difference.


**Research involving human participants and/or animals:** This study was approved by the Institutional Animal Care and Use Committee of the Changchun University of Chinese Medicine. We have strictly carried out the relevant research work protecting the rights and interests of animals under the supervision of the Institutional Animal Care and Use Committee to ensure that the research is in line with the relevant provisions of the Institutional Animal Care and Use Committee.
**Informed consent:** Informed consent was obtained from all individual participants included in the study.
**Ethics approval:** All applicable international, national and/or institutional guidelines for the care and use of animals were followed.
**Data availability statement:** The analyzed data sets generated during the present study are available from the corresponding author on reasonable request.

## 3 Results

### 3.1 circ_AKT3 level is upregulated and miR-206 level is downregulated in cisplatin-resistant GC

To probe the role of circ_AKT3 and miR-206 in cisplatin resistance, their levels were detected in cisplatin-sensitive or resistant GC tissues. Compared with sensitive samples (*n* = 42), circ_AKT3 level was evidently enhanced in cisplatin-resistant GC tissues (*n* = 23) (Figure 1a). On the contrary, the abundance of miR-206 was abnormally reduced in resistant tissues in comparison to that in sensitive group (Figure 1b). Moreover, the data from Figure 1c and d displayed that IC_50_ of cisplatin in MKN-7/DDP and HGC-27/DDP cells was higher than that in MKN-7 and HGC-27 cells, which suggested the high resistance of both MKN-7/DDP and HGC-27/DDP cells to cisplatin. The data of RT-qPCR assay showed that circ_AKT3 expression was obviously increased in MKN-7/DDP and HGC-27/DDP cells in comparison to sensitive cells, while miR-206 abundance showed an opposite trend (Figure 1e and f). The above data suggested that cisplatin resistance might be associated with circ_AKT3 and miR-206.

**Figure 1:** circ_AKT3 expression is elevated and miR-206 level is decreased in resistant GC. (a and b) The levels of circ_AKT3 and miR-206 were measured in sensitive (*n* = 42) and resistant (*n* = 23) GC tissues via RT-qPCR. (c and d) The IC_50_ of cisplatin was analyzed in MKN-7, MKN-7/DDP, HGC-27 and HGC-27/DDP cells by MTT assay. (e and f) The levels of circ_AKT3 and miR-206 were detected in DDP-sensitive and DDP-resistant GC cells via RT-qPCR. *P < 0.05.

### 3.2 Interference of circ_AKT3 reduces cisplatin resistance in resistant GC cells

To assess the biological role of circ_AKT3 in cisplatin resistance, circ_AKT3 was silenced in MKN-7/DDP and HGC-27/DDP cells by a siRNA. As displayed in Figure 2a, circ_AKT3 expression was effectively reduced in MKN-7/DDP and HGC-27/DDP cells after transfection of si-circ_AKT3, showing the high efficiency of si-circ_AKT3 in reducing circ_AKT3 expression. MTT assay displayed that circ_AKT3 knockdown significantly decreased the IC_50_ of cisplatin in the two cell lines (Figure 2b). Moreover, downregulation of circ_AKT3 inhibited the expression of P-gp protein level in MKN-7/DDP and HGC-27/DDP cells (Figure 2c and d). In addition, the analysis of flow cytometry showed higher apoptotic rate in the two resistant cell lines after silencing circ_AKT3 as compared with the two sensitive cell lines (Figure 2e and f). The above findings manifested that circ_AKT3 knockdown improved sensitivity of GC cells to cisplatin.

**Figure 2:** Silence of circ_AKT3 inhibits cisplatin resistance of resistant GC cells. MKN-7/DDP and HGC-27/DDP cells were transfected with si-circ_AKT3 or s-NC. Then, circ_AKT3 expression (a), IC_50_ of cisplatin (b), P-gp protein level (c and d) and apoptosis (e and f) were measured via RT-qPCR, MTT, Western blot and flow cytometry, respectively. *P < 0.05.

### 3.3 Overexpression of miR-206 represses cisplatin resistance of resistant GC cells

The role of miR-206 in cisplatin resistance was also explored in MKN-7/DDP and HGC-27/DDP cells by overexpressing miR-206 using miRNA mimic. After the transfection of miR-206 mimic, miR-206 abundance was markedly increased in MKN-7/DDP and HGC-27/DDP cells (Figure 3a). Then, miR-206 overexpression induced obvious reduction in IC_50_ of cisplatin in the two types of resistant cells (Figure 3b). Meanwhile, the results of Western blot demonstrated that miR-206 overexpression led to a decline in P-gp protein production (Figure 3c and d). Besides, the apoptotic rate of MKN-7/DDP and HGC-27/DDP cells was significantly increased by miR-206 overexpression (Figure 3e and f). Taken together, these results explained that miR-206 was able to improve cisplatin sensitivity in GC cells.

**Figure 3:** Overexpression of miR-206 suppresses cisplatin resistance of resistant GC cells. The expression of miR-206 (a), IC_50_ of cisplatin (b), P-gp protein level (c and d) and apoptosis (e and f) were detected in MKN-7/DDP and HGC-27/DDP cells with transfection of miR-206 mimic or miR-NC via RT-qPCR, MTT, Western blot and flow cytometry, respectively. *P < 0.05.

### 3.4 circ_AKT3 regulates cisplatin resistance of resistant GC cells by sponging miR-206

Results of bioinformatics analysis displayed that circ_AKT3 carried the complementary sites of miR-206 (Figure 4a), suggesting the potential correlation between them. To validate this interaction, the Wt or Mut luciferase reporter vectors of circ_AKT3 were constructed and transfected into MKN-7/DDP and HGC-27/DDP cells. Results first showed that miR-206 overexpression induced decrease in luciferase activity in circ_AKT3-Wt-transfected cells, but the luciferase activity of circ_AKT3-Mut had no response to miR-206 overexpression (Figure 4b and c). Moreover, RNA pull-down assay revealed the binding ability of circ_AKT3 and miR-206 by biotinylated miR-206 or circ_AKT3, respectively (Figure 4d and e). According to spearman’s correlation analysis, miR-206 expression in GC tissues was inversely associated with circ_AKT3 level (*r* = −0.629 and *P* < 0.001) (Figure 4f). Subsequently, the effect of circ_AKT3 on miR-206 level was investigated in MKN-7/DDP and HGC-27/DDP cells by overexpressing or silencing circ_AKT3. As exhibited in Figure 4g and h, miR-206 abundance was obviously inhibited by circ_AKT3 overexpression, but enhanced by circ_AKT3 interference. To explore whether the effect of circ_AKT3 on cisplatin resistance was modulated via miR-206, MKN-7/DDP and HGC-27/DDP cells were transfected with si-NC, si-circ_AKT3, si-circ_AKT3 + anti-miR-NC or anti-miR-206. The data of RT-qPCR demonstrated that transfection of anti-miR-206 obviously abolished the promoting impact of circ_AKT3 interference on miR-206 expression level (Figure 5a). Besides, the rescue experiments displayed that miR-206 deficiency attenuated the inhibitive role of circ_AKT3 silence in IC_50_ of cisplatin and P-gp protein level as well as the promoting effect of circ_AKT3 on apoptosis (Figure 5b–f). Thus, all these findings explained that circ_AKT3 regulated cisplatin resistance by interacting with miR-206 in GC cells.

**Figure 4:** circ_AKT3 is a decoy of miR-206. (a) The potential complementary sites of circ_AKT3 and miR-206 were analyzed via starBase. (b and c) Luciferase activity was detected in MKN-7/DDP and HGC-27/DDP cells co-transfected with miR-NC or miR-206 mimic and circ_AKT3-Wt or circ_AKT3-Mut. (d and e) The levels of circ_AKT3 and miR-206 were detected in MKN-7/DDP and HGC-27/DDP cells after biotin pull-down. (f) The linear correlation between expression of circ_AKT3 and miR-206 in GC tissues was analyzed. (g and h) miR-206 level was detected in MKN-7/DDP and HGC-27/DDP cells transfected with vector, circ_AKT3 overexpression vector, si-NC or si-circ_AKT3 via RT-qPCR. *P < 0.05.

**Figure 5:** Down-regulation of miR-206 attenuates the effect of circ_AKT3 knockdown on cisplatin resistance of resistant GC cells. MKN-7/DDP and HGC-27/DDP cells were transfected with si-NC, si-circ_AKT3, si-circ_AKT3 + anti-miR-NC or anti-miR-206. Then, miR-206 level (a), IC_50_ of cisplatin (b), P-gp protein level (c–e) and apoptotic rate (f) were investigated by RT-qPCR, MTT, Western blot and flow cytometry, respectively. *P < 0.05.

### 3.5 miR-206 inhibits cisplatin resistance of resistant GC cells via targeting PTPN14

The mRNA and protein levels of PTPN14 were evidently enhanced in cisplatin-resistant GC tissues and cells (Figure 6a–d). Meanwhile, PTPN14 level was negatively associated with miR-206 level in GC tissues (Figure 6e). To further elucidate the mechanism, bioinformatics analysis showed that miR-206 was able to bind to PTPN14 (Figure 6f). Subsequent results displayed that the luciferase activity was notably reduced in PTPN14 3′UTR-Wt + miR-206 group in MKN-7/DDP and HGC-27/DDP cells, but it was not changed in PTPN14 3′UTR-Mut + miR-206 group (Figure 6f). Moreover, restoration of PTPN14 weakened the effect of miR-206 overexpression on IC_50_ of cisplatin, P-gp expression and cell apoptosis in MKN-7/DDP and HGC-27/DDP cells (Figure 6g–i). By large, all the above observations demonstrated that PTPN14 could regulate cisplatin resistance through interaction with miR-206.

**Figure 6:** miR-206 inhibits cisplatin resistance of resistant GC cells via targeting PTPN14. (a and b) PTPN14 expression was measured in sensitive (*n* = 42) and resistant (*n* = 23) GC tissues via RT-qPCR and Western blot. (c and d) PTPN14 expression was detected in sensitive and resistant GC cells by RT-qPCR and Western blot. (e) The linear correlation between levels of PTPN14 and miR-206 in GC tissues was analyzed. (f) The binding sites of miR-206 and PTPN14 were searched via starBase, and luciferase activity was detected in MKN-7/DDP and HGC-27/DDP cells co-transfected with miR-NC or miR-206 mimic and PTPN14 3′UTR-Wt or PTPN14 3′UTR-Mut. IC_50_ of cisplatin (g), P-gp protein level (h) and apoptotic rate (i) were measured in MKN-7/DDP and HGC-27/DDP cells transfected with miR-NC, miR-206 mimic, miR-206 mimic + pcDNA or PTPN14 overexpression vector via MTT, Western blot and flow cytometry, respectively. *P < 0.05.

### 3.6 circ_AKT3 modulates PTPN14 expression by miR-206

To explore whether circ_AKT3 could regulate PTPN14 in DDP-resistant GC cells, MKN-7/DDP and HGC-27/DDP cells were transfected with si-NC, si-circ_AKT3, si-circ_AKT3 + anti-miR-NC or anti-miR-206. As displayed in Figure 7a–c, PTPN14 expression at mRNA and protein levels were notably decreased via knockdown of circ_AKT3, which were restored by inhibition of miR-206, indicating that circ_AKT3 regulated PTPN14 by associating with miR-206.

**Figure 7:** circ_AKT3 regulates PTPN14 expression via miR-206 in resistant GC cells. (a–c) PTPN14 expression was detected in MKN-7/DDP and HGC-27/DDP cells transfected with si-NC, si-circ_AKT3, si-circ_AKT3 + anti-miR-NC or anti-miR-206 via RT-qPCR and Western blot. *P < 0.05.

### 3.7 circ_AKT3 knockdown decreases xenograft tumor growth

The study continued to explore the effect of circ_AKT3 *in vivo*. As shown in Figure 8a and b, the volume and weight of tumors were obviously declined in sh-circ_AKT3 group in comparison to sh-NC group. In addition, circ_AKT3, PTPN14 and P-gp levels were reduced and miR-206 abundance was increased in tumor samples from sh-circ_AKT3 group in comparison to sh-NC group (Figure 8c–e). The above data ascertained that circ_AKT3 knockdown inhibited MKN-7/DDP cell malignancy *in vivo*.

**Figure 8:** Knockdown of circ_AKT3 reduces xenograft tumor growth. MKN-7/DDP cells stably transfected with sh-circ_AKT3 or sh-NC were used for establishment of xenograft model. (a) Tumor volume was detected every 4 days. (b) Weight of tumor tissues was measured at the end point. (c–e) The levels of circ_AKT3, miR-206, PTPN14 and P-gp were detected in each group. *P < 0.05.

## 4 Discussion

Previous studies demonstrated that circRNAs could act as miRNA sponges or competing endogenous RNAs (ceRNAs) to further modulate drug resistance in GC [20,21]. Moreover, it was reported that circ_AKT3 contributed to cisplatin resistance in GC [9]. Nevertheless, more insights in the mechanism of circ_AKT3 regulating cisplatin resistance in GC are needed. In the current research, circ_AKT3 was highly expressed in GC tissues and cells with cisplatin resistance. Knockdown of circ_AKT3 decreased cisplatin resistance by downregulating P-gp expression. For the first time, we demonstrated a ceRNA network of circ_AKT3/miR-206/PTPN14 that was associated with cisplatin resistance.

In this study, we found high level of circ_AKT3 might be associated with cisplatin resistance in GC, indicating the positive role of circ_AKT3 in GC, which was opposite to that in other cancers [7,8]. We hypothesized that the exact roles of circRNAs in cancers might be induced due to the alteration of tumor microenvironment. By using MKN-7/DDP and HGC-27/DDP cells, we found that silencing circ_AKT3 decreased cisplatin resistance as reduction in IC_50_ of cisplatin and increase in apoptosis after circ_AKT3 knockdown, which was consistent with the findings of previous study [9]. P-gp is one of the key proteins associated with drug resistance and can trigger multidrug resistance in GC [22,23]. This study found that circ_AKT3 knockdown inhibited P-gp protein expression in GC, suggesting the inimical role of circ_AKT3 in chemotherapy. The ceRNA regulatory network, including circRNA, miRNA and mRNA, is one of the main mechanisms associated with tumorigenesis and pathogenesis of GC [24]. To explore whether circ_AKT3 regulated cisplatin resistance by functioning as a ceRNA, its potential target miRNAs were searched. As a result, we confirmed circ_AKT3 acted as a sponge for miR-206 in GC cells.

miR-206 has been reported to negatively modulate drug resistance in human cancers [11,12,13,14]. In the current work, low level of miR-206 was involved in cisplatin resistance and its overexpression attenuated the cisplatin resistance by regulating P-gp. This was also consistent with previous studies [14,15]. Moreover, the effect of circ_AKT3 silence on cisplatin resistance was weakened by miR-206 exhaustion, indicating that circ_AKT3 regulated drug resistance by sponging miR-206 in GC. To further explore the ceRNA crosstalk of circ_AKT3, the target mRNA of miR-206 was searched. Previous studies focusing on the role of miR-206 in human cancers have showed some targets, such as cyclinD2, CXC chemokine receptor 4 and mitogen activating protein kinase 3 (MAPK3) [15,25,26]. This research validated PTPN14 as a functional target of miR-206 using luciferase reporter analysis.

Previous studies suggested PTPN14 served as an oncogene in GC by regulating proliferation, migration and epithelial-to-mesenchymal transition [16,27,28]. Moreover, PTPN14 was implicated in paclitaxel and doxorubicin resistance in GC [17]. Our study showed that PTPN14 expression was elevated in cisplatin-resistant GC, indicating that PTPN14 might also contribute to cisplatin resistance. Furthermore, we found that PTPN14 weakened the effect of miR-206 on cisplatin resistance, and it was regulated by circ_AKT3 through miR-206. Collectively, circ_AKT3 induced PTPN14 to participate in the regulation of cisplatin resistance by sponging miR-206 in GC cells. To better understand the underlying mechanism, *in vivo* experiments were performed. And our data confirmed the suppressive effect of circ_AKT3 knockdown on growth of cisplatin-resistant GC cells *in vivo*.

## 5 Conclusion

In conclusion, our findings described the sensitization role of circ_AKT3 knockdown in GC, uncovered by decrease in IC_50_ of cisplatin and P-gp expression and increase in apoptosis. The inner mechanism was that circ_AKT3 regulated miR-206/PTPN14 axis in a ceRNA-based manner. This work first confirmed the ceRNA network of circ_AKT3/miR-206/PTPN14, providing a new idea for ameliorating cisplatin sensitivity in GC treatment.

## Abbreviations

anti-miR-206: miR-206 inhibitor
anti-miR-NC: miR-206 inhibitor negative control
circRNAs: circular RNAs
circ_AKT3: circRNA AKT serine/threonine kinase 3
GC: gastric cancer
IC_50_
: half maximal inhibitory concentration
miRNAs: microRNAs
miR-NC: miRNA negative control
P-gp: p-glycoprotein
TPN14: protein tyrosine phosphatase non-receptor type 14
si-NC: siRNA for negative control
siRNA: small interfering RNA
RT-qPCR: quantitative reverse transcription PCR
vector: pcDNA circRNA mini vector
